# Acute Erythemal Ultraviolet Radiation Causes Systemic Immunosuppression in the Absence of Increased 25-Hydroxyvitamin D_3_ Levels in Male Mice

**DOI:** 10.1371/journal.pone.0046006

**Published:** 2012-09-26

**Authors:** Shelley Gorman, Naomi M. Scott, Daryl H. W. Tan, Clare E. Weeden, Robert C. Tuckey, Jacqueline L. Bisley, Michele A. Grimbaldeston, Prue H. Hart

**Affiliations:** 1 Telethon Institute for Child Health Research and Centre for Child Health Research, University of Western Australia, Perth, Western Australia, Australia; 2 School of Biomedical, Biomolecular and Chemical Sciences, University of Western Australia. Perth, Western Australia, Australia; 3 Division of Human Immunology, Centre for Cancer Biology, SA Pathology, Adelaide, South Australia, Australia; Nihon University School of Medicine, Japan

## Abstract

Vitamin D is synthesised by ultraviolet (UV) irradiation of skin and is hypothesized to be a direct mediator of the immunosuppression that occurs following UV radiation (UVR) exposure. Both UVR and vitamin D drive immune responses towards tolerance by ultimately increasing the suppressive activities of regulatory T cells. To examine a role for UVR-induced vitamin D, vitamin D_3_-deficient mice were established by dietary vitamin D_3_ restriction. In comparison to vitamin D_3_-replete mice, vitamin D_3_-deficient mice had significantly reduced serum levels of 25-hydroxyvitamin D_3_ (25(OH)D_3_, <20 nmol.L^−1^) and 1,25-dihydroxyvitamin D_3_ (1,25(OH)_2_D_3_, <20 pmol.L^−1^). Following either acute erythemal UVR, or chronic sub-erythemal UVR (8 exposures over 4 weeks) treatment, serum 25(OH)D_3_ levels significantly increased in vitamin D_3_-deficient female but not male mice. To determine if UVR-induced vitamin D was a mediator of UVR-induced systemic immunosuppression, responses were measured in mice that were able (female) or unable (male) to increase systemic levels of 25(OH)D_3_ after UVR. Erythemal UVR (≥4 kJ/m^2^) suppressed contact hypersensitivity responses (T helper type-1 or -17), aspects of allergic airway disease (T helper type-2) and also the *in vivo* priming capacity of bone marrow-derived dendritic cells to a similar degree in female and male vitamin D_3_-deficient mice. Thus, in male mice, UVR-induced 25(OH)D_3_ is not essential for mediating the immunosuppressive effects of erythemal UVR.

## Introduction

UV irradiation of skin causes a systemic immunosuppression in both humans and mice [1]. Much is still unknown about the mechanisms that control systemic immunity following UV irradiation [2]. Postulated immune mediators of UV radiation (UVR)-regulated systemic immunosuppression include soluble products released by skin cells like keratinocytes and mast cells, altered antigen presenting cell precursors at distant sites like the bone marrow and UVR-induced regulatory T and B cells (reviewed in [3], [4]). A potential immune regulator induced by UVR is vitamin D_3_. For humans, much of our vitamin D_3_ is obtained from processes consequent to the absorption of UVB photons by 7-dehydrocholesterol in skin [5]. The active form of vitamin D_3_, 1,25(OH)_2_vitamin D_3_ (1,25(OH)_2_D_3_), is then produced both locally by keratinocytes [6], and systemically by successive hydroxylations in the liver and kidney. Post-UV irradiation (or dietary intake), serum levels of the metabolite 25-hydroxyvitamin D_3_ (25(OH)D_3_) are used as a measure of vitamin D status.

In a recent review, we analysed whether vitamin D may be responsible for the immunosuppression that occurs after UVR [3]. UV irradiation damages the DNA of skin-resident dendritic cells (DC) [7], [8] and induces their migration into the skin-draining lymph nodes [8]. These DCs then increase the suppressive activity and/or numbers of lymph node-resident CD4+CD25+Foxp3+ regulatory T cells [8]–[10]. Similarly, topical application of 1,25(OH)_2_D_3_ induces migration of skin DCs into the draining lymph nodes [11] to control regulatory T cells [11], [12]. UVR [13] and topical calcipotriol (a vitamin D analog, [11]) both induce RANKL expression by keratinocytes, which in turn stimulate the expansion of antigen-specific regulatory T cells. These observations support a model of UVR-induced local immunosuppression (at the skin site that receives UVR) that is mediated through 1,25(OH)_2_D_3_ with downstream effects on keratinocytes, dendritic cells and regulatory T cells.

To date, investigations of UVR have not examined immune responses in vitamin D-deficient individuals. Indeed, the role of UVR-induced vitamin D in modulating immune-driven diseases has not (until the current study) been examined in vitamin D-deficient mice. Through dietary restriction, vitamin D deficiency enhanced the pathogenesis of immune-driven disorders such as diabetes [14], colitis [15] and arthritis [16] in rodent models. However, Becklund et al (2010), observed that UVR suppressed experimental autoimmune encephalomyelitis (EAE) in mice (a murine model of multiple sclerosis) when there were minimal changes in serum 25(OH)D_3_, suggesting that vitamin D_3_ may not be a central mediator of UVR-induced systemic immunosuppression [17].

In the current study, we used a novel approach to examine a role of UVR-induced vitamin D_3_ in suppressing systemic immune responses in murine models of contact hypersensitivity (CHS, T helper type-1/17 cell-mediated) and allergic airway disease (T helper type-2 cell-mediated). By provision of specially designed diets with or without vitamin D_3_, mice became vitamin D_3_-replete or -deficient, respectively. Mice were exposed to a single acute erythemal dose of UVR, or to chronic suberythemal UVR. After UV irradiation, significantly increased serum 25(OH)D_3_ levels were recorded only in female mice that were initially vitamin D_3_-deficient. Male vitamin D_3_-deficient mice consistently did not respond to UVR with no increases detected in serum 25(OH)D_3_ levels. We then evaluated immune responses in mice that were able (female) or unable (male) to synthesize vitamin D to evaluate a role for UVR-induced vitamin D in UVR-induced systemic immunosuppression.

## Materials and Methods

### Mice and Diet

All experiments were performed according to the ethical guidelines of the National Health and Medical Research Council of Australia and with approval from the Telethon Institute for Child Health Research Animal Ethics Committee. Mice were purchased from the Animal Resources Centre, Western Australia. Female 3 wk-old BALB/c mice were placed on semi-pure diets which were (SF05-34, Specialty Feeds, Perth, Western Australia, 1% Ca^2+^) or were not (SF05-033, Specialty Feeds, 2% Ca^2+^) supplemented with 2280 IU vitamin D_3_/kg. At 8 weeks of age, female mice were mated with adult male BALB/c mice maintained on standard mouse chow (Specialty Feeds). Offspring born following these matings were maintained on the vitamin D_3_-replete or -deficient diets for the rest of the experiment. In some experiments BALB/c or C57Bl/6 mice were placed on the vitamin D_3_-replete or -deficient diets from 4 weeks of age. Mice were housed under perspex-filtered fluorescent lighting, which emitted no detectable UVB radiation as measured using a UV radiometer (UVX Digital Radiometer, Ultraviolet Products Inc., Upland, CA, USA).

### Measurement of Serum Vitamin D and Calcium Levels

Levels of 25(OH)D_3_ and 1,25(OH)_2_D_3_ levels were measured in serum and/or ear tissue lysates [18] using IDS EIA ELISA kits (Immunodiagnostic Systems Ltd, Fountain Hills, AZ) as described by the manufacturer. Ear lysates were prepared as previously described by Biggs et al (2010) for quantification of 1,25(OH)_2_D_3_ levels 24 h after skin exposure to UVR [18]. 1,25(OH)_2_D_3_ levels were adjusted to account for the diluting effects of edema which occurs 24 h after exposure of skin to erythemal UVR. For confirmation, 25(OH)D_3_ levels in selected samples were measured using the DiaSorin Liaison method (Saluggia, Italy) and by isotope-dilution liquid chromatography-tandem mass spectrometry by RMIT Drug Discovery Technologies (Melbourne, Australia). Calcium levels in serum were determined by the Vitros dry chemistry method (Vitros 250, Ortho Clinical Diagnostics, Raritan, NJ).

### UV Radiation

A bank of six 40 W lamps (Philips TL UV-B, Eindhoven, The Netherlands) emitting broadband UVR, 250–360 nm, with 65% of the output in the UVB range (280–315 nm), was used to irradiate mice to deliver various doses of UVR onto clean-shaven 8 cm^2^ dorsal skin as previously described [19], [20]. A new sheet of PVC plastic film (0.22 mm) was taped to the top of each perspex cage immediately before irradiation to screen wavelengths <280 nm. Sunlamps were held 20 cm above the cages. Unless used in CHS experiments, the ears were not covered or taped for the UV treatments.

### Measurement of 7-dehydrocholesterol Levels in Skin

Shaved dorsal skin (1 cm^2^) was removed from mice and snap-frozen in liquid N_2_. 7-dehydrocholesterol was extracted from 0.1 g of the frozen skin by homogenization with 4 ml CHCl_3_/CH_3_OH 1∶1 (v/v) as described for cholesterol extraction [21]. 7-dehydrocholesteol esters present in the extract were hydrolysed with sodium methoxide and then quantitated by HPLC as previously described [22], except that a C18 column (Kinetex 5 cm × 4.6 mm particle size 2.6 µm) was used with samples being applied in 80% methanol and eluted with a 80–100% methanol gradient in water (25 min) followed by 100% methanol (15 min) at a flow rate of 0.5 ml/min. 7-dehydrocholesterol was detected with a UV monitor at 280 nm.

### Detection of mRNA

Messenger mRNA was extracted from the kidneys of naïve 8 week-old vitamin D_3_-replete or -deficient mice with cDNA synthesized and real-time assays performed as previously described [12], [20] using Quantitect Primer Assays (Qiagen, Doncaster, VIC, Australia) for detection of CYP27B1 and CYP24A1 with EEF1α used as the house-keeping control [12].

### CHS Responses

A CHS assay was performed using 2,4-dinitrofluorobenzene (DNFB, Sigma Chemical Company, St Louis, MO) as previously described [20], [23]. Mice were sensitized by painting 25 µl 0.5% DNFB diluted in acetone onto the shaved ventral surface. After another 5 days, a CHS response was elicited by painting dorsal and ventral ear surfaces with 10 µl 0.2% DNFB (in acetone). After 24 hours, the ear thickness was measured in a blinded manner spring-loaded micrometer (Mitutoyo Corp, Aurora, IL) as described previously [19]. In all experiments, some mice were challenged but not sensitized with 0.2% DNFB (in acetone).

### Measurement of Edema in UV-irradiated Skin

At various times post-UV irradiation, the double skin thickness of back skin was measured using a spring-loaded micrometer at 3 locations, 1 cm apart, across the back. These measurements were averaged and the pre-UV irradiation reading subtracted.

### Measuring the in vivo Priming Capacity of Bone Marrow-derived DCs (BMDCs)

DCs were expanded *in vitro* from the bone marrow of mice harvested 3 days after UV irradiation. CD11c+ cells were purified from the loosely adherent bone marrow cells resulting after 7 days culture with GM-CSF and IL-4 as previously described [24]. The cells were loaded with dinitrobenzenesulfonic acid-sodium salt prior to subcutaneous injection of 10^6^ cells into the ear pinnae of naïve (vitamin D_3_-replete) mice. Dinitrobenzenesulfonic acid-sodium salt is a water-soluble analogue of DNFB. Cells were obtained from and injected into mice of the same sex. Seven days later, each ear pinnae of the recipient mice was challenged with 10 µl DNFB (0.2% in acetone), and ear-swelling responses measured 24 h after this challenge using a spring-loaded micrometer.

### Bronchoalveolar Lung Lavage of Mice Sensitized and Challenged with Ovalbumin

OVA (Sigma) in alum (Serva, Heidelberg, Germany) was delivered i.p. on day 0 (10 µg OVA in 2 mg alum per mouse; 200 µl volume) and again on day 14. Mice were then challenged on days 21, 22 and 23 with a 1% OVA-in-saline aerosol delivered using an ultrasonic nebulizer (UltraNebs, DeVilbiss, Somerset, PA) for 30 min [25]. Twenty-four hours after the final aerosol, BALF was collected as described previously [25]. BALF cells were then centrifuged onto slides and stained using the DIFF-Quik Stain Set 64851 (Lab Aids, Narrabeen, NSW, Australia) as per the manufacturer’s instructions. Levels of IL-5 in BALF were detected using ELISA as previously described [25].

### Statistical Analyses

Data were compared using an unpaired two-way student’s *t* test using the Prism 5 for Mac OS X statistical analysis program as appropriate.

## Results

### Generating Vitamin D_3_-replete and -deficient Mice

Dietary manipulation was used to generate vitamin D_3_-deficient and -replete mice [26]. BALB/c female mice were fed vitamin D_3_-containing (replete) or -null diets from 3 weeks of age. Upon weaning offspring born to these female mice were continued on the restricted diet of their mother. At 8 weeks of age (adulthood), the offspring mice raised on the diets that were or were not supplemented with vitamin D_3_ were of equal weight and size, and had mean serum levels of 25(OH)D_3_ of >50 nmol.L^−1^ and <20 nmol.L^−1^, respectively (Figure 1A) [26]. As observed previously, male mice fed the vitamin D_3_-replete diet had significantly lower serum levels of 25(OH)D_3_ than female mice fed the same diet (Figure 1A) [26]. Levels of the further hydroxylated form, 1,25(OH)_2_D_3_ were significantly lower in the serum of vitamin D_3_-“deficient” mice compared with -“replete” mice as observed previously [15], although there was no difference in levels observed between female and male mice (Figure 1B). There was no difference in the serum calcium levels recorded for mice on either diet (Figure 1C).

**Figure 1:** Dietary vitamin D_3_ restriction reduces serum 25(OH)D_3_ and 1,25(OH)_2_D_3_ levels. Female BALB/c mice were placed on vitamin D_3_ (VitD)-containing or -deficient diets from 3 weeks of age. At 8 weeks of age the female mice were mated with adult BALB/c male mice (fed vitamin D_3_-replete diets). In (A), (B) and (C), serum 25(OH)D_3_, 1,25(OH)_2_D_3_ and calcium levels (respectively) were measured in female and male 8 week-old offspring of these matings (n = 5 mice/group). In (D), 7-dehydrocholesterol levels were determined in the skin of vitamin D_3_-deficient female and male mice. In (E), kidney CYP27B1 mRNA levels induced by vitamin D_3_ deficiency in female and male mice are shown. In (F), kidney CYP27B1 and CYP24A1 mRNA levels induced by being male for vitamin D_3_-replete (VitD+) and -deficient (VitD-) mice. For (A)–(F), data is shown as mean + SEM, with n≥3 mice/group, *p<0.05 between groups, #p<0.05 relative to levels in vitamin D3-replete (E) or female (F,G) mice.

### Male Vitamin D_3_-deficient Mice have Reduced Skin Levels of the Vitamin D Precursor, 7-dehydrocholesterol

Levels of the vitamin D_3_ precursor, 7-dehydrocholesterol, were significantly lower in the skins of vitamin D_3_-deficient male than female mice when mice were tested at 8 weeks of age (Figure 1D). In the kidneys, vitamin D_3_ deficiency per se enhanced CYP27B1 mRNA levels above levels observed in vitamin D_3_- replete animals for both female and male mice (Figure 1E). CYP27B1 is the 25-hydroxyvitamin D_3_ 1α-hydroxylase that hydroxylates 25(OH)D_3_ to form 1,25(OH)_2_D_3_ [3], [5]. Male vitamin D_3_-replete and -deficient mice also expressed increased levels of CYP27B1 mRNA than female vitamin D_3_-replete and -deficient mice, respectively (Figure 1F). Male vitamin D_3_-deficient mice expressed 3-fold more CYP24A1 mRNA in the kidneys than female -deficient mice (Figure 1F), but this was not observed in the vitamin D_3_-replete mice. CYP24A1 encodes an enzyme responsible for initiating degradation of 1,25(OH)_2_D_3_ [3], [5].

### Vitamin D Status in Male Vitamin D_3_-deficient Mice is Unaltered by UVR

Serum levels of 25(OH)D_3_ in vitamin D_3_-replete mice did not significantly change from those depicted in Figure 1A in response to acute erythemal (8 kJ/m^2^) or chronic sub-erythemal UV irradiation (8 exposures to ≤2 kJ/m^2^ UVR over 4 weeks)(data not shown). However, in vitamin D_3_-deficient mice, significant increases in serum 25(OH)D_3_ levels were measured in the female but not the male mice in response to a single dose of 4 or 8 kJ/m^2^ UVR (Figure 2A). In female vitamin D_3_-deficient mice a significant increase was detected in response to a single exposure of 2 kJ/m^2^ UVR but not 1 kJ/m^2^ UVR, 4 and 11 days after irradiation (Figure 2B), although serum levels remained <25 nmol.L^−1^. In response to chronic low dose UVR (1 or 2 kJ/m^2^) administered 8 times over 4 weeks, serum 25(OH)D_3_ levels increased in female but not male vitamin D_3_-deficient mice (Figure 2C). When 8-week old female and male vitamin D_3_-deficient mice were fed the vitamin D_3_-supplemented diet for 4 weeks, all mice increased their serum 25(OH)D_3_ levels to >50 nmol.L^−1^ (Figure 2D). As observed previously (Figure 1A) [26], male mice fed the vitamin D_3_-supplemented diet had significantly lower serum 25(OH)D_3_ in comparison to female mice (Figure 2D). These levels were comparable to those observed in mice fed the vitamin D_3_-supplemented diet from conception until adulthood (Figure 1A) [26]. In comparison to 4 week-old (post-weaning, pre-pubescent) female mice, 4 week-old male mice also failed to produce significant serum 25(OH)D_3_, 7 days after irradiation with 4 kJ/m^2^ UVR (Figure 2E). Serum calcium levels of female and male vitamin D_3_-deficient mice did not change when measured 7 days after 8 kJ/m^2^ UVR (Figure 2F). Vitamin D_3_-replete 4-week old BALB/c (Figure 2G) or C57Bl/6 (Figure 2H) mice were fed a vitamin D_3_-deficient diet for 28 days prior to UV irradiation (8 kJ/m^2^). Only the female mice responded to UV exposure with significantly increased serum 25(OH)D_3_ levels, 7 days post-UVR. Thus, the inability of male mice to alter the serum 25(OH)D_3_ levels after UVR was not dependent on whether they had been maintained on a vitamin D_3_-containing diet since conception.

**Figure 2:** UVR enhances 25(OH)D_3_ levels in the serum of vitamin D_3_-deficient female but not male mice. The shaved dorsal surfaces of eight week-old female and male offspring of vitamin D_3_-deficient female BALB/c mice were irradiated with either (A) a single dose of 4 or 8 kJ/m^2^ UV (n ≥4 mice/group, *p<0.05 for female versus male), or (B) females were irradiated with 1 or 2 kJ/m^2^ UV (*p<0.05 for 1 versus 2 kJ/m^2^ UV). After 1, 4, 7 and/or 11 days, serum 25(OH)D_3_ levels were measured. In (C), vitamin D_3_-deficient offspring were chronically irradiated with 1 or 2 kJ/m^2^ UV at the times indicated by arrows and serum 25(OH)D_3_ levels monitored (n = 3 mice/group, *p<0.05 for female versus male). In (D), vitamin D_3_-deficient offspring were placed on the vitamin D_3_-replete diet and serum 25(OH)D_3_ levels assessed over 30 days (n = 8 mice/group, *p<0.05 for all times versus 0 days). In (E), 4 week-old vitamin D_3_-deficient mice were irradiated with 4 kJ/m^2^ UV, with serum 25(OH)D_3_ levels measured 7 days post-irradiation (n = 3 mice/group, *p<0.05). In (F), serum calcium levels were determined in female and male vitamin D_3_-deficient mice 7 days after 8 kJ/m^2^ UV irradiation (n = 6 mice/group). In (G) and (H), 4 week-old vitamin D_3_-replete BALB/c or C57Bl/6 mice were fed a vitamin D_3_-deficient diet for 28 days before UV irradiation (8 kJ/m^2^), respectively. After a further 7 days, serum 25(OH)D_3_ levels were measured (n = 5 mice/group, *p<0.05 for female versus male). For (A)–(D), (G) and (H), data are shown as mean ± SEM, and for (E) and (F), data are shown as mean + SEM.

### 1,25(OH)_2_D_3_ Levels Increase in the Skin of Vitamin D_3_-replete Females but not Males 24 h after Acute Erythemal UVR

Keratinocytes express the full repertoire of enzymatic machinery required for the conversion of 7-dehydrocholesterol into active 1,25(OH)_2_D_3_ following UV irradiation of skin [27]. Vitamin D_3_-replete or -deficient BALB/c mice were exposed to 8 kJ/m^2^ and the levels of 1,25(OH)_2_D_3_ assessed 24 h later in UV-irradiated ear skin. Increased 1,25(OH)_2_D_3_ levels were observed in ear skin lysates of vitamin D_3_-replete female, but not male mice (Figure 3A). In addition, no change in 1,25(OH)_2_D_3_ levels was detected in the ear skin of either male or female vitamin D_3_-deficient mice with UV irradiation (Figure 3A). UVR (8 kJ/m^2^) also did not significantly alter serum 1,25(OH)_2_D_3_ levels at 4 days post-irradiation (Figure 3B), which remained significantly reduced in the serum of the vitamin D_3_-deficient mice relative to the -replete controls (Figure 3B).

**Figure 3:** Erythemal UVR does not increase 1,25(OH)_2_D_3_ in the skin and serum of vitamin D_3_-deficient mice. Levels of 1,25(OH)_2_D_3_ were assessed in the (A) skin and (B) serum of vitamin D_3_-replete (VitD) or -deficient female or male BALB/c mice exposed to 0 or 8 kJ/m^2^ UVR. In (A), 1,25(OH)_2_D_3_ were assessed in the ear skin of mice (n = 6 ears/treatment) 24 h after UVR. In (B), 1,25(OH)_2_D_3_ were assessed in the serum of mice (n≥4 mice/treatment) 96 h after UVR. For (A) and (B), data is shown as mean + SEM, *p<0.05 between groups.

### Can UVR Suppress CHS Responses in Vitamin D_3_-deficient Mice when Antigen is Applied to a Skin Site Distant to that UV-irradiated?

A CHS assay provides a measure of a T helper type-1/17-driven immune response and has been frequently used to study UVR-induced immune suppression in both humans and mice [28], [29]. The “systemic” immunosuppressive effects of UVR were examined in vitamin D_3_-deficient female and male BALB/c mice by delivering UVR to the shaved dorsal skin of mice 4 days before the exposure of ventral skin to the sensitizer, DNFB. In separate experiments, 4 or 8 kJ/m^2^ UVR significantly suppressed the CHS response in both the female and male vitamin D_3_-deficient mice to a similar degree (Figure 4A). To evaluate the extent of the UVR insult, vitamin D_3_-deficient and -replete mice were administered different doses of UVR and the induced edema measured. Both UVR doses were edemal, but importantly the edema was not altered by vitamin D_3_ deficiency (Figure 4B for results in male mice, data not shown for female mice). As observed previously [19]–[20], [23], UVR (≥4 kJ/m^2^) suppressed systemic CHS ear-swelling responses in female or male vitamin D_3_-replete mice by ∼50% (data not shown). We observed no difference in the CHS responses in the vitamin D_3_-replete or -deficient mice (data not shown). In addition, UV-induced lymph node hypertrophy [20], [23] was measured in the auricular lymph nodes (ALN) of vitamin D_3_-deficient mice irradiated with 0 or 8 kJ/m^2^ UV (Figure 4C). The number of ALN cells per mouse was increased by a similar extent in both female and male mice, 4 days post-UV irradiation. In summary, UVR suppressed CHS responses in vitamin D_3_-deficient males in a systemic fashion when antigen was applied to a non-irradiated site, and enhanced skin edema and LN hypertrophy, in the absence of changes to circulating 25(OH)D_3_ levels (Figure 2).

**Figure 4:** UVR suppresses CHS responses to a similar degree in female and male (initially) vitamin D_3_-deficient mice, when antigen was applied to a skin site distal to the UV-irradiated site. In (A), ear thickness after the sensitization and challenge of BALB/c mice with DNFB. Results shown were combined from four experiments in which the shaved dorsal skins of mice were irradiated with 4 (2 experiments) or 8 kJ/m^2^ UV (2 experiments). Mice were sensitized through the ventral skin with DNFB, 4 days after UV irradiation, and ears challenged 4 days later with ear swelling measured after a further 24 h. In (A), results from female and male mice are depicted as open and closed bars, respectively. In (B), the double skin-fold thickness of dorsal skin of vitamin D_3_-replete (solid lines) and vitamin D_3_-deficient (broken lines) male mice after irradiation with 4 or 8 kJ/m^2^ UV irradiation is shown at various times for a representative experiment (of 3 performed). In (C), the number of ALN cells per mouse is shown 4 days after irradiation of (unprotected) ears with 4 kJ/m^2^ UV. For (A) and (C), results are shown as mean + SEM and data in (B) is shown as mean ± SEM (*p<0.05, n = 4 mice/treatment/experiment).

### Can UVR Suppress CHS Responses in Vitamin D_3_-deficient Mice when Antigen is Applied to the UV-irradiated Site?

The immunosuppressive effects of UVR were also examined locally by delivering UVR (8 kJ/m^2^) to the shaved dorsal skin of vitamin D_3_-deficient mice, 4 days before application of DNFB to the same dorsal skin site. UVR significantly suppressed “local” CHS responses in both the female and male vitamin D_3_-deficient mice to a similar extent (Figure 5A).

**Figure 5:** UVR suppresses immune responses in female and male (initially) vitamin D_3_-deficient mice. (A) CHS responses when antigen was applied to the UV-irradiated site. Ear thickness after the sensitization and challenge of BALB/c mice with DNFB is shown. Shaved dorsal skins of mice were irradiated with 8 kJ/m^2^ UV. Mice were sensitized through the dorsal skin with DNFB (4 days after UV irradiation) and ears challenged 4 days later with ear swelling measured after a further 24 h. (B) BMDCs from UV-irradiated female or male vitamin D_3_-deficient mice have impaired *in vivo* priming abilities. Female and male vitamin D_3_-deficient BALB/c mice were irradiated with 8 kJ/m^2^ UVR. Three days later, DCs were expanded by culturing bone marrow cells from the non-irradiated and UV-irradiated mice for 7 days with GM-CSF and IL-4. Isolated CD11c+ cells were loaded with dinitrobenzenesulfonic acid-sodium salt and then injected epicutaneously into the ears of naïve mice. After a further 7 days, the ears of recipient mice were challenged with DNFB and ear swelling measured 24 h later. For both (A) and (B), ear thickness measurements are shown as mean + SEM (*p<0.05, n = 4 mice/treatment), with results from female and male mice depicted as open and closed bars, respectively.

### UVR Reduces the in vivo Priming Ability of Bone Marrow-derived DCs from Vitamin D_3_-deficient Female and Male Mice to a Similar Extent

BMDCs from UV-irradiated mice have an impaired ability to prime immune responses *in vivo* [24]. To examine the systemic effect of UVR in vitamin D_3_-deficient mice, DCs were expanded *in vitro* from the bone marrow of UV-irradiated mice and used to prime a CHS response in naïve (and sex-matched) mice. UVR significantly suppressed the capacity of BMDCs (CD11c+ cells) from female and male vitamin D_3_-deficient mice to prime T helper type-1/17 ear-swelling responses in recipient mice to a similar extent (Figure 5B). These results suggest that the capacity of UVR to modify DC precursors in the bone marrow is independent of circulating levels of 25(OH)D_3_ post-UV irradiation.

### ‘Low’ Dose UVR Significantly Increases Serum 25(OH)D_3_ Levels without Suppressing Local Immune Responses

To further differentiate the outcomes of UVR and increased serum 25(OH)D_3_ levels, three daily doses of 2 kJ/m^2^ UVR [8] were administered to the dorsal skin of female vitamin D_3_-deficient BALB/c mice before applying DNFB to dorsal skin 24 h after the final UV irradiation (Figure 6A). Multiple 2 kJ/m^2^ doses of UVR raised serum 25(OH)D_3_ levels to >50 nmol.L^−1^ in female mice (Figure 6A). This UVR regime did not suppress ear-swelling responses in the irradiated BALB/c mice (Figure 6B) to a ‘locally’-applied antigen (DNFB), even though mice were sensitized when serum levels of 25(OH)D_3_ had significantly increased post-UVR (Figure 6A). These observations again confirm that the ability of UVR to modulate serum 25(OH)D_3_ is independent of its capacity to suppress immune responses in the strains of mice tested.

**Figure 6:** Three doses of 2 kJ/m^2^ UVR increases serum 25(OH)D_3_ but does not suppress CHS in female (initially) vitamin D_3_-deficient mice. The shaved dorsal skin of female vitamin D_3_-deficient BALB/c mice was irradiated (or not) with three daily doses of 2 kJ/m^2^ UVR (+ UV). Mice were sensitized through the dorsal skin with DNFB (4 days after UV irradiation) and ears challenged 4 days later. Ear swelling measured after a further 24 h. In (A), serum 25(OH)D_3_ levels were determined 24 h after the final UV irradiation, and 24 h after ear-challenge. In (B), ear thickness measurements are shown. Data is shown in (A) as mean ± SEM and in (B) as mean + SEM (n = 4 mice/treatment, *p<0.05 for + UV versus − UV).

### Effect of UVR on Allergic Airway Responses in Vitamin D_3_-deficient Mice

We have previously shown that erythemal UV irradiation (≥2 kJ/m^2^) of skin reduces asthma-like pathologies in two murine models of allergic airways disease [25], [30]. To determine the contribution of vitamin D_3_ towards regulating allergic airway disease after UV irradiation, vitamin D_3_-deficient female or male mice were UV-irradiated (8 kJ/m^2^), or not, 3 days before sensitization with ovalbumin (OVA) with the adjuvant, alum. The extent of allergic airways disease was examined 24 h after the final respiratory challenge with OVA. In each of three independent experiments, sensitization to OVA was greater in the female than male vitamin D_3_-deficient mice (Figure 7). This was shown in the non-irradiated mice, where more eosinophils (Figure 7A) and increased IL-5 levels (Figure 7B) were detected in the BALF of the female mice. For results combined from three experiments, the number of eosinophils (Figure 7A) and the levels of IL-5 (Figure 7B) in the BALF were significantly reduced by UV irradiation of the female and male mice that were initially vitamin D_3_-deficient. After normalization to remove the variation in sensitization observed between the female and male mice, there was no difference in the extent of UVR-induced suppression of eosinophil numbers (Figure 7C) or IL-5 concentrations (Figure 7D) in the BALF observed in the female and male mice. Thus, in the absence of UVR-induced increases in serum 25(OH)D_3_ in the male vitamin D_3_-deficient mice, UVR significantly suppressed T helper type-2-specific responses (eosinophilia and IL-5 in lavage fluid) in this model of allergic airway disease.

**Figure 7:** UVR suppresses asthma-like Th2 responses to a similar degree in female and male (initially) vitamin D_3_-deficient mice. Vitamin D_3_-deficient female or male BALB/c mice were UV irradiated (8 kJ/m^2^) and three days later were sensitized and boosted with OVA and alum on days 0 and 14, respectively. On days 21, 22 and 23 mice were challenged with an OVA aerosol. After a further 24 h, bronchoalveolar lavage fluid was obtained. In (A), eosinophil numbers, and in (B), IL-5 concentrations in the bronchoalveolar lavage fluid are shown. In (C) and (D), eosinophil numbers and IL-5 concentrations were normalized relative to eosinophils numbers and IL-5 concentrations measured for non-irradiated OVA-sensitized, -boosted and -challenged mice to remove the effects of gender on allergic sensitization. The mean result from each experiment was used to calculate the results shown (mean + SEM, n = 3 experiments, *p<0.05, n = 4 mice/group/experiment), with results from female and male mice depicted as open and closed bars, respectively.

## Discussion

In this study, male vitamin D_3_-deficient mice were unable to increase their serum 25(OH)D_3_ levels in response to UVR, in contrast to female mice. Even though serum 25(OH)D_3_ levels did not change after UV treatment of male mice, the capacity of a single erythemal dose of UVR to suppress immune responses was very similar in male and female vitamin D_3_-deficient mice. Multiple immune models (CHS and allergic airway disease) were used to show that UVR-induced immunosuppression was independent of serum levels of 25(OH)D_3_. A variety of substances produced by skin cells aside from vitamin D_3_ may control UVR-induced systemic immunosuppression [3], [4]. For example, UV irradiation of skin acts at least partially through prostanoids to reduce the immune priming ability of BMDCs [24]. Furthermore, after erythemal UVR, prostaglandin E_2_ signals through the EP4 receptor to increase regulatory T cell numbers through enhanced epidermal RANKL expression [31]. While further work is required to characterize the immune pathways responsible for the systemic immunosuppression caused by UVR, we now present evidence that UVR-induced vitamin D may not be essential for immunosuppression.

UVR did not increase serum 25(OH)D_3_ levels in either BALB/c or C57Bl/6 vitamin D_3_-deficient male mice, suggesting that this effect is not strain-dependent. This defect is not detrimental to the general health of male mice as while they are mainly nocturnal and covered in fur, and they have evolved an efficient system to obtain vitamin D_3_ from their food and not skin exposure to sunshine. Our studies and those of others [5], suggest that synthesis of vitamin D_3_ by UVR in the skin of vitamin D_3_-deficient mice occurs by the same processes in mice as for humans. We propose that reduced levels of the precursor 7-dehydrocholesterol in the skin of male versus female mice (summarized in Figure 8) contributes significantly towards the inability of male mice to produce serum 25(OH)D_3_ after UV irradiation but are uncertain as to why male mice have less 7-dehydrocholesterol than females. Other mammals exhibit very low or undetectable quantities of 7-dehydrocholesterol in their skin, including cats and dogs [22]. In humans, the extent of variation of cutaneous 7-dehydrocholesterol levels is not known. In patients with dietary malabsorption disorders like Crohn’s disease, 7-dehydrocholesterol levels are increased in their skin relative to age- and sex-matched control subjects [32]. This interesting finding does indicate that there may be regulatory links between vitamin D metabolism in the skin and gut, but these need further investigation. Age reduces 7-dehydrocholesterol levels in human skin [33]. As UVR did not increase 25(OH)D_3_ levels in 4 week-old pre-pubescent male mice, their modulation by UVR in female mice only is likely to be independent of hormonal status.

Other non-skin-related defects in vitamin D metabolism exist in male mice as serum levels of 25(OH)D_3_ were lower in male mice fed a vitamin D_3_-replete diet relative to the female animals. In addition, the expression of the 1,25(OH)_2_D_3_ synthesis and breakdown enzymes (CYP27B1 and CYP24A1, respectively) in the kidneys were upregulated in male, relative to female vitamin D_3_-deficient mice suggesting that 1,25(OH)_2_D_3_ metabolism and catabolism may occur at a faster rate in male mice, as suggested by others [34]. Even so, male and female vitamin D_3_-deficient mice had similarly reduced serum levels of 1,25(OH)_2_D_3_, relative to their -replete counterparts, as observed previously [15]. The extent of ear swelling induced by a CHS assay was comparable in male and female mice using the hapten dinitrofluorobenzene (eg. Figure 4A). Others have also reported that the capacity of UVB irradiation to modulate CHS responses is equivalent in male and female (vitamin D-replete) mice [35], [36] but describe gender differences in UV-induced inflammation and immunosuppression in response to exposure to UVA radiation (315–400 nm) [36]. It is the UVB wavelengths of sunlight that are responsible for converting 7-dehydrocholesterol into pre-vitamin D in the skin [5], and are of most relevance for the current studies.

**Figure 8:** Vitamin D deficiency modifies the expression of key molecules of the vitamin D metabolic pathways differently in male and female mice. A summary of the synthesis of 1,25(OH)_2_D_3_ from 7-dehydrocholesterol in skin in relation to the observed effects on this pathway following UV-irradiation of vitamin D_3_-deficient female and male mice. Post-UVR changes in 25(OH)D_3_ and 1,25(OH)_2_D_3_ levels are depicted by arrows with no change shown as (−).

In the vitamin D_3_-deficient mice, we did not observe significant synthesis of 1,25(OH)_2_D_3_ in skin 24 h after exposure to erythemal UVR, which suppressed both systemic and local CHS responses in the vitamin D_3_-deficient mice. These results suggest that the ability of erythemal UVR to suppress immunity may be independent of cutaneous synthesis of 1,25(OH)_2_D_3_. However, a role for 1,25(OH)_2_D_3_ in modulating immunity after chronic sub-erythemal UVR is plausible. Indeed, local skin inflammation induced by chronic sub-erythemal UVR may be controlled by mast cells and their response to UVR-induced 1,25(OH)_2_D_3_ [18]. Inflammation induced by chronic UVR (2 kJ/m^2^, 15 doses over 30 days) was enhanced in the skin of mast cell-deficient mice (WBB6F_1_-Kit^W/Wv^) that were engrafted with bone marrow-derived mast cells from VDR^−/−^ mice relative to wild-type controls [18]. These studies suggest that the VDR may be important for the ability of mast cells to suppress skin inflammation caused by sub-erythemal UVR. It is therefore possible that 1,25(OH)_2_D_3_ may be an important mediator that controls local skin immune responses after chronic sub-erythemal but not erythemal doses of UVR. In addition, many different immune cells, including dendritic cells can synthesize 1,25(OH)_2_D_3_ to potentially modulate local immunity [3]. However, we anticipate that low levels of circulating 25(OH)D_3_ may reduce the capacity of such cells to synthesize 1,25(OH)_2_D_3_ to regulate immunity, especially in male mice, where UVR alone cannot modify serum 25(OH)D_3_ levels.

UV irradiation of skin can be beneficial in the treatment of not only hypersensitivity responses and models of asthma, but also models of multiple sclerosis [37], and by inference other diseases characterized by hyperimmune reactivity. This study complements an examination of UV control of EAE in mice [17]. UV irradiation of skin reduced the expression of the disease but as the mice used were not vitamin D_3_-deficient, there were minimal measurable changes in serum 25(OH)D_3_ levels. As previously published [38], the EAE disease model can be regulated by a diet containing 1,25(OH)_2_D_3_, and to a lesser extent by a diet containing very high levels of 25(OH)D_3_. The diet containing the 1,25(OH)_2_D_3_ stimulated significant hypercalcaemia which, rather than the vitamin D_3_ *per se*, may regulate EAE development [38]. In contrast, UVR reduced EAE symptoms in mice but calcium levels did not change [17].

In this study, we have used a physiological model of vitamin D_3_-deficiency and not VDR or CYP27B1 knockout mice to investigate a role for vitamin D in mediating UV-induced immunosuppression. There are many problems associated with using mice with the VDR or CYP27B1 gene knocked out globally, or even in a tissue-specific manner. Both VDR^−/−^ and CYP27B1^−/−^ mice have serious developmental problems that lead to dermatological, skeletal, reproductive and immune dysfunction [5]. For adequate bone development and survival, VDR^−/−^ knockout mice need to be fed a rescue diet consisting of 2% Calcium and 20% Lactose [39]. VDR^−/−^ mice also have alopecia and exhibit keratinocyte stem cell defects [5]. CYP27B1^−/−^ mice do not have alopecia, but their keratinocytes exhibit reduced expression of differentiation markers and have an inhibited ability to recover normal skin barrier function after an acute perturbation [5]. The alopecia observed in the VDR^−/−^ mice is independent of 1,25(OH)_2_D_3_ expression. We anticipate that these ligand-independent effects would still occur in the skin of mice with keratinocyte-specific knockdown of expression of the VDR. Other studies indicate that the VDR acts as a tumour suppressor independently of 1,25(OH)_2_D_3_. VDR^−/−^ mice exhibit reduced rates of thymine-dimer repair and apoptosis in UV-exposed skin and these dysfunctional epidermal repair pathways coincided with an enhanced susceptibility to the development of skin tumours induced by chronic UV irradiation or by a chemical carcinogen [40]. In a recent paper, normal bone phenotype in CYP27B1^−/−^ mice was partially restored by treating the knockout mice with vitamin D_3_ [41]. In particular, body weight and bone-related parameters were restored by chronic intramuscular treatment with 10,000 IU vitamin D_3_/week for 4 weeks [41]. These effects were mediated in the absence of conversion to 1,25(OH)_2_D_3_, where 25(OH)D_3_ may be another albeit lower-affinity ligand of the VDR. These studies suggest that CYP27B1^−/−^ mice can still respond to vitamin D, and are thus an incomplete model to study the effects of ‘vitamin D deficiency’ on disease. Finally, results observed in vitamin D_3_-deficient mice are not always found in VDR^−/−^ mice. For example, a reduced asthma phenotype occurs in VDR^−/−^ mice [42] while asthma severity is enhanced in vitamin D_3_-deficient mice [26] and inhibited in mice treated with 1,25(OH)_2_D_3_ [43]–[45]. Together, these findings using VDR^−/−^ and CYP27B1^−/−^ mice further highlight how the development and regeneration of the skin (and other tissues) of these knockout mice is dependent on the expression of the VDR (and perhaps also CYP27B1), and indicate that they are not suitable (or physiologically relevant) models for investigating the effects of UVR on skin immunity.

Our physiologically-relevant studies show that male vitamin D_3_-deficient mice are unable to make 25(OH)D_3_ in response to UVR when deficiency was induced only by removal of vitamin D_3_ from the diet. The levels of 25(OH)D_3_ observed in the mice on the vitamin D_3_-null diet mimic the cut-offs for vitamin D deficiency (<25 nmol.L^−1^) suggested for humans [3]. The source of vitamin D_3_ for these deficient mice with low, but detectable serum 25(OH)D_3_ levels is unknown, but may be due to a naturally-occurring contaminant of the wheat starch component of the non-vitamin D_3_-supplemented diet. Our findings have significant health implications. We demonstrate that the potential benefits of UVR in reducing the morbidity associated with systemic immune disorders such as asthma or multiple sclerosis, may not be dependent on circulating levels of 25(OH)D_3_, as particularly observed in male mice. Based on the experimental models tested, we observed that vitamin D synthesis is not required for systemic (or local) immunosuppression after erythemal UVR. In conclusion, this study suggests that while the benefits of UV irradiation of skin and vitamin D_3_ supplementation in modulating inappropriate systemic immune responses may be complementary, vitamin D synthesis is not essential for mediating the immunosuppressive effects of UVR.
